# Hypothalamus-adipose tissue crosstalk: neuropeptide Y and the regulation of energy metabolism

**DOI:** 10.1186/1743-7075-11-27

**Published:** 2014-06-10

**Authors:** Wei Zhang, Mark A Cline, Elizabeth R Gilbert

**Affiliations:** 1 3200 Litton-Reaves, Animal & Poultry Sciences Department, Virginia Tech, Blacksburg, VA 24061-0306, USA

**Keywords:** Adipose tissue, Hypothalamus, neuropeptide Y, Obesity, Sympathetic nervous system, Thermogenesis

## Abstract

Neuropeptide Y (NPY) is an orexigenic neuropeptide that plays a role in regulating adiposity by promoting energy storage in white adipose tissue and inhibiting brown adipose tissue activation in mammals. This review describes mechanisms underlying NPY’s effects on adipose tissue energy metabolism, with an emphasis on cellular proliferation, adipogenesis, lipid deposition, and lipolysis in white adipose tissue, and brown fat activation and thermogenesis. In general, NPY promotes adipocyte differentiation and lipid accumulation, leading to energy storage in adipose tissue, with effects mediated mainly through NPY receptor sub-types 1 and 2. This review highlights hypothalamus-sympathetic nervous system-adipose tissue innervation and adipose tissue-hypothalamus feedback loops as pathways underlying these effects. Potential sources of NPY that mediate adipose effects include the bloodstream, sympathetic nerve terminals that innervate the adipose tissue, as well as adipose tissue-derived cells. Understanding the role of central vs. peripherally-derived NPY in whole-body energy balance could shed light on mechanisms underlying the pathogenesis of obesity. This information may provide some insight into searching for alternative therapeutic strategies for the treatment of obesity and associated diseases.

## Introduction

Obesity is defined as a state of increased adiposity resulting from chronic nutrient excess, where energy intake significantly exceeds energy expenditure [1]. Energy intake is reflected by food intake and energy expenditure can be affected by basal metabolism, physical activity, and thermogenesis [2]. Dysregulation of either central or peripheral signals may lead to a state of anorexia or obesity. According to the Center for Disease Control in 2011–2012, more than one third of all U.S. adults are considered to be overweight or obese and these numbers are expected to continue to rise. The rise in obesity, a predisposing factor for developing diabetes, hypertension, hyperlipidemia, cancer and other disorders, has driven a major interest in the regulation of appetite, food intake and fat accumulation [3]. Energy homeostasis is governed by a complex neuroendocrine system including appetite regulatory hypothalamic peptides, as well as adipocyte-derived peripheral signals such as leptin. These signals act in a reciprocal manner to integrate information about energy status, a system referred to as the hypothalamus-adipose tissue axis. The recognition of the importance of the hypothalamus-adipose tissue axis in energy balance has propelled studies aimed at understanding the roles of adipose- and hypothalamic-derived peptides on energy intake, storage and expenditure.

One of the major regulators of energy intake, neuropeptide Y (NPY), has emerged as an important player in the hypothalamus-adipose tissue axis. Neuropeptide Y, a 36 amino acid peptide, is one of the most potent orexigenic hypothalamic neuropeptides identified to date [4]. Depending on the anatomical location and the receptor sub-type, NPY is also involved in other physiological processes such as locomotion, learning and memory, anxiety, epilepsy, circadian rhythm, and cardiovascular function [3]. The goal of this review is to provide a more in-depth and holistic understanding of the role of NPY in energy homeostasis, bridge the gap between appetite/central nervous system and adipose tissue/peripheral studies, as well as define current challenges and possible future study directions. To emphasize the potential dual roles of NPY in energy intake and energy storage/expenditure, we highlight the idea of hypothalamus and adipose tissue crosstalk and the connection to the sympathetic nervous system. Numerous studies demonstrate that NPY is a major mediator in promoting energy storage, positing that it could serve as a potential biomarker for obesity. Consistent with this hypothesis, the NPY receptor sub-type 5 (NPYR5) antagonist, velneperit, has been recently explored in clinical testing as a potential anti-obesity drug [5]. Therefore, a better understanding of the mechanisms of how NPY influences body adiposity may facilitate therapeutic interventions for obesity.

### NPY and receptor sub-type tissue distribution

In the central nervous system (CNS), NPY is found in highest concentration within the hypothalamus, brain stem, and anterior pituitary. In the arcuate nucleus (ARC) of the hypothalamus, NPY is highly expressed with another orexigenic neuropeptide, agouti-related peptide (AgRP), an endogenous melanocortin receptor 3 and 4 (MC3R and MC4R, respectively) antagonist [6]. The ARC NPY neurons serve as a feeding center that senses and integrates peripheral energy signals, such as blood glucose concentration, ghrelin, leptin and insulin, due to the unique anatomic structure of the ARC in lacking a blood brain barrier [7]. The synthesis and secretion of ARC NPY is induced in response to energy deficiency and greater metabolic demand such as increased exercise, cold and pregnancy [8].

The NPY affects food intake by innervating with other appetite regulatory factors in the CNS and regulates energy utilization via modulation of fat deposition and metabolism. These functions are achieved by binding to various NPY receptors (NPYRs) that are distributed across the body, the most well-known being NPYR1, NPYR2, and NPYR5, all of which are G protein coupled receptors [9]. In situ hybridization assays on adult mouse brain sections revealed widespread distribution of NPYR1, while NPYR2 and 5 displayed a more restricted pattern of expression [10]. The NPYR1 is considered to be most directly involved in food intake and energy expenditure, whereas the NPYR2 receptor is an autoreceptor that is mainly expressed in the ARC, and can regulate food intake and energy balance through modulation of endogenous NPY release [11,12]. The NPYR1 has a high affinity for the NPY analog [Leucine^31^, Proline^34^] and requires a complete N terminus for binding. It has lower affinity for NPY C-terminal fragments such as NPY_13–36_ and NPY_3–36_[13]. The NPYR2 requires intact carboxyl-terminal fragments for binding [14]. The preferred binding ligands, distribution of NPYRs, and NPY function in the CNS and adipose tissue are summarized in Table 1.

**Table 1:** Neuropeptide Y family receptors with preferred ligands, receptor distribution and function in food intake and fat deposition

		**Y1**	**Y2**	**Y4**	**Y5**
**Preferred ligand**		**NPY**	**NPY**	**PP**	**NPY**
		**Requires a complete N terminus**	**NPY3-36**	**NPY**	**NPY2-36**
			**Requires intact C-terminal fragments**		**NPY3-36**
Pre vs. post junctional receptor		Post-junctional	Pre-junctional	Post-junctional	Post-junctional
Distri-bution	Brain (besides hypotha-lamus)	Cortex, brainstem, hippocampus, thalamus, amygdala	Cortex, brainstem, hippocampus, amygdala, striatum, nucleus accumbens	Subnucleus gelatinosus of NTS, dorsal motor nucleus of the vagus	Cortex, hippocampus, amygdala
	Hypoth-alamus	ARC, VMN, PVN, DMN, LH Supraoptic nucleus	ARC, PVN, LH, medial preoptical area, anterior hypothalamic nucleus	ARC, PVN	PVN, ARC, VMN, DMN, LH
	Perip-heral	Thyroid, parathyroid glands, heart, spleen and digestive system, adipose tissue	Adipose tissue	Skeletal muscle, small intestine, pancreas, prostate, uterus, lung, colon	Adipose tissue
Types of manipulation/Effects on food intake and body weight		Y1 antagonist central injection/Reduced food intake [15,16]; Y1 agonist central injection/Increase food intake [17]; Y1KO/Developed obesity, increased body fat, slight reduction in food intake [18,19]	Y2 agonist IP injection/ inhibit food intake [20]; Hypothalamus-specific Y2 KO/Increased food intake and decreased body weight; Germ-line Y2 KO/Reduced body weight and adiposity, reduced food intake in males and increased food intake in females [21]	Y4 KO/Decreased body weight, less WAT, decreased 24-h food intake in male mice [22]	Central administration of Y5 antisense oligodeoxynucleotides/Reduced body weight and a decrease in food intake [23,24]; Y5 KO/ Mild late-onset obesity, increased body weight, food intake and adiposity [25]

Abbreviations: *KO* knock out, *NTS* Nucleus of the solitary tract, *WAT* white adipose tissue, *ARC* arcuate nucleus, *PVN* Paraventricular nucleus, *VMN* ventromedial nucleus, *DMN* dorsomedial nucleus, *LH* Lateral hypothalamic area, *IP injection* intraperitoneal injection. Other references used for this table besides the papers cited above [13,26-28]. The references are not exhaustive but rather indicate key initial and/or representative studies.

In the periphery, NPY is widely distributed in the sympathetic nerves, the adrenal medulla, platelets, and various cell types within white adipose tissue [26]. The expression of NPY and NPYR2 can be induced in macrophages [29], platelets, nerves, and adipocytes by stress or genetically- or high fat diet-induced obesity in mice [29,30]. In human adipose tissue, NPY was detected in mature adipocytes but not in preadipocytes [31]. Others detected NPY mRNA in human subcutaneous and visceral fat [32] and murine adipocytes as well as various cell types from adipose tissue stromal vascular fractions (SVF) [29]. Increased expression of NPY in adipose tissue appears to be a common feature of obesity in different species. Abundance of NPY mRNA and protein was greater in visceral fat (pooled mesenteric, omental and retroperitoneal) of 21 day-old obese rats born from dams that were fed a low-protein diet during gestation and lactation, compared to controls [33]. There was also greater NPY mRNA in visceral fat of obese Zucker rats compared to their lean counterparts, and both an insulin analogue and dexamethasone augmented NPY expression in lean but not obese rats [33]. We reported greater expression of NPY and NPYR1 and NPYR5 mRNA in the abdominal fat of obese chickens compared to lean chickens [34].

The NPYR1, NPYR2 and NPYR5 have all been detected in various cell types from different fat depots in rodent models [29,35,36], although in one report NPYR5 was not detected by real time PCR in either adipocytes or the SVF of adipose tissue from either lean or obese mice [29] and in another only NPYR5 was detected in sympathetic neuron/3 T3-L1 co-cultures [37]. Human and mouse preadipocytes, adipocytes and endothelial cells express NPYR2 [30] and mouse NPYR1 expression was detected in mouse preadipocytes and adipocytes [37]. Others reported that NPYR1 mRNA was abundant in both rat and mouse preadipocytes, whereas NPYR2 and NPYR5 were undetectable [33]. We demonstrated that NPY, NPYR1, NPYR2 and NPYR5 mRNA were expressed in chicken abdominal fat, albeit at lower quantities than in the hypothalamus, with differential expression between chickens selected for low or high body weight, and highly negative heterosis, suggesting a role for the NPY system in energy balance in chickens [34]. Thus, in a variety of vertebrates, NPY and NPYR1, 2 and 5 are expressed in various cell types in white adipose tissue.

### Adipose tissue function and sympathetic nervous system innervation

As the primary energy storage reservoir, adipose tissue plays an important role in energy balance. It contains two distinct types of fat tissue: white adipose tissue (WAT) and brown adipose tissue (BAT). White adipose tissue is specialized for the storage of chemical energy in the form of triacylglycerol (TAG), while BAT dissipates chemical energy in the form of heat through non-shivering thermogenesis. As will be discussed in this review, major mechanisms for WAT expansion and turnover are changes in rates of adipocyte precursor cell proliferation, differentiation of precursor cells into adipocytes (adipogenesis), as well as changes in synthesis of fatty acids (lipogenesis), TAGs, and hydrolysis of stored lipids (lipolysis) to liberate glycerol and free fatty acids in the adipocyte [38]. Unlike WAT, BAT dissipates chemical energy in the form of heat generation by means of uncoupling protein 1 (UCP1) expression to uncouple respiration in the mitochondria [2]. Increased BAT in animals was associated with a lean and healthy phenotype [39], whereas loss of BAT was correlated with obesity and metabolic diseases [40]. BAT is predominantly distributed in the interscapular region of mammals. Although brown fat was once considered only necessary in early neonates, recent positron emission tomography scanning studies demonstrated that this tissue is present and plays a pivotal role in energy balance in adult humans [41,42]. Therefore, induction of BAT in humans offers the possibility of increasing energy expenditure without necessarily causing dysfunction in other tissues, and is hence an obvious therapeutic target for treating obesity.

White adipose tissue is a heterogeneous organ comprised of mature adipocytes, preadipocytes, mesenchymal stem cells, immune cells, and a matrix of collagen fibers that house numerous nerve endings and vascular networks [43]. Thus, NPY can potentially affect WAT metabolism through the neuroendocrine route, where it is co-stored with norepinephrine (NE) and can be secreted via sympathetic nervous system (SNS) innervation, autocrine mechanisms by mature adipocytes, paracrine pathways by immune cells [29], as well as endocrine routes by platelets from the blood vessels, or across the blood brain barrier [44]. Neuropeptide Y coexists within the nerve terminal with NE and adenosine triphosphate in postganglionic sympathetic nerve fibers throughout the body, and can be co-released from the axon terminals in different quantities depending on the stimulation intensity and the pattern of sympathetic nerve activation [45,46]. Retrograde and anterograde fluorescence tract tracers were used to reveal sympathetic innervation of adipose tissue and that different fat depots were differentially innervated (reviewed by [47]). As will be described later in this review, the hypothalamus-SNS-WAT pathway provides a plausible mechanism for how NPY exerts reciprocal functions on energy intake via the hypothalamus and energy storage and expenditure via WAT.

### NPY promotes adipogenesis and inhibits lipolysis in adipose tissue

NPY was shown to have hyperplasic, adipogenic and antilipolytic effects in adipose tissue cells, and angiogenic effects in the vasculature surrounding adipose cells (a major contributor to adipose expansion) both in vitro and in vivo [30,48], although in one study there was no effect of NPY treatment on lipid accumulation in 3 T3-L1 cells at 8 days post-differentiation [33]. Effects of NPY on adipose tissue function were thought to occur mainly via NPYR1- and NPYR2-mediated pathways, although NPYR5 has also been implicated in the cellular responses [14,30,44,49,50]. Two weeks of cold exposure, combined with consumption of a high-fat and high-sugar diet, was associated with increased expression of NPY and NPYR2 in subcutaneous fat depots of mice, with expression localized to blood vessels, nerves and adipocytes [30]. Conditional knockdown of NPYR2 in only the peripheral tissues (including adipose) of adult mice prevented high fat diet-induced obesity [51]. In normal chow-fed mice, the knockdown had no effect on food intake or body weight, suggesting that NPYR2 plays an important role in energy oxidation in peripheral tissues [51]. The NPYR2 germline knock-out mice were not susceptible to cold stress-induced augmentation of diet-induced obesity and treatment of wild-type mice with a NPYR2 antagonist for 2 weeks via slow-release pellets delivered to the adipose tissue reduced visceral fat depot mass by 40%. Similarly, conditional knockdown of NPYR2 by an adenoviral vector injected into the subcutaneous abdominal fat of mice led to a 50% reduction in stress-induced fat expansion after 2 weeks [30]. These results collectively suggest that those NPY-mediated effects on adipose tissue were occurring mainly through NPYR2 [30]. Similarly, in immune-deficient mice or rhesus monkeys that received subcutaneous injections of a 14-day slow-release NPY pellet, a ring of new fat tissue appeared around the pellet, and was sustained for at least 3 months, demonstrating the ability of NPY to locally promote de novo fat formation [52]. Neuropeptide Y-mediated effects on fat were also demonstrated with a translational application to reconstructive surgery [52]. Freshly collected human adipose tissue was transplanted into immune-deficient mice and effects of NPY on fat graft survival and vascularity were assessed [52]. Treatment with NPY enhanced long-term (3 month) human fat graft survival and vascularity in the athymic mice, whereas in mice that did not receive NPY pellet injection, there was greater than 70% resorption of the xenograft, a major concern with such transplantation surgeries in humans [52]. Researchers showed that the effects on fat pad mass were due to enhanced survival of the human graft and not synthesis of new adipose tissue by the host animal, illustrating a potential clinical application of NPY.

In genetically obese (B6.V-Lep^ob/J^) mice, plasma concentrations of NPY were more than 200% greater than wild-type mice, and the obese mice also displayed greater expression of NPY and NPYR2 mRNA in subcutaneous fat, suggesting that the elevated circulating NPY originated from adipose tissue [30]. Interestingly, in both obese and lean wild-type mice, there was substantial adipose tissue expansion as a result of treatment with NPY pellets (1 μg per 14-day release pellet) delivered locally to the subcutaneous abdominal fat [30]. These effects were blunted when mice were injected with a pellet containing BIIE0246, an NPYR2 antagonist (1 umol/day for 14 d), with a decrease in fat mass accompanied by reduced vascularity and increased apoptosis in the abdominal fat pads [30]. Results from these studies implied that NPY’s actions on adipose tissue include promotion of both adipogenesis and angiogenesis, both mediated primarily through NPYR2 [30].

Function through NPYR2 could be mediated through enzymatic cleavage of the NPY peptide in adipose tissue [48]. In one study, NPY and dipeptidyl peptidase –IV (DPPIV) mRNA were detected in both 3 T3-L1 preadipocytes and terminally differentiated adipocytes, and treatment of preadipocytes with recombinant DPPIV promoted differentiation of cells into adipocytes [48]. The DPPIV is known to cleave NPY into the NPYR2 agonist NPY_3–36_. Immunoneutralization of NPY or treatment with a NPYR2 antagonist, but not NPYR1 or NPYR5 antagonists, blunted DPPIV’s adipogenic effects [48]. Treatment with NPY alone also promoted preadipocyte differentiation and combined treatment of NPY with a DPP-IV inhibitor , vildagliptin, blocked NPY’s adipogenic effects, lending further support to the idea that DPP-IV cleaves NPY in adipose tissue and thereby promotes adipogenesis via NPYR2-mediated cell signaling [48].

Effects of NPY on TAG hydrolysis, on the other hand, were shown to occur mainly through NPYR1, with effects on lipolysis influenced by the nutritional state, other cellular factors, and genetic background of the animal. For example, in cultured rat adipocytes, NPY dose-dependently inhibited lipolysis, an effect that was blunted when the animals were fasted for 48 hours prior to treatment [14]. Receptor-specific NPY fragments were used to show that inhibition of lipolysis was mediated through NPYR1. In visceral fat cells (but not subcutaneous) from rats that were injected with 6-hydroxydopamine (OHDA) (a neurotoxin for sympathetic neurons that is used to chemically ablate sympathetic nerves), lipolysis was increased and the effects were shown to occur via NPYR2-mediated signaling mechanisms [14]. Using receptor-specific peptide fragments, it was shown that inhibition of lipolysis in adipose tissue occurred through NPYR1 but not NPYR2, and that the increase in lipolysis observed after sympathectomy and treatment with a NPYR2-specific peptide could be due to a switching of the receptor from G_i_ to G_s_ coupling [14].

Metabolic differences observed between subcutaneous and visceral fat depots may be partly explained by differences in SNS innervation. In general, visceral fat in humans is associated with adverse health outcomes, whereas subcutaneous adipose tissue is considered to be an energy storage reservoir that is relatively benign [38]. Recently, Nguyen et al. demonstrated that while there was some overlap in central sympathetic neural circuits between inguinal (subcutaneous) and mesenteric (visceral) fat in Siberian hamsters, there were more neurons involved in innervating the inguinal fat pads, and interestingly, food withdrawal induced a stronger sympathetic drive to inguinal adipose tissue [53]. Thus, research on NPY’s role in adipose tissue function should take into consideration the differences in physiology between fat depots in different anatomical locations under different nutritional conditions.

The effects of NPY on lipolysis appear to be highly dependent on other cellular factors influencing β-adrenergic stimulation in the adipocyte. In one study, NPY was shown to have no effect on lipolysis in differentiated 3 T3-L1 cells under basal conditions, but augmented β-adrenergic-mediated stimulation of lipolysis [54]. When cells were pretreated with isoproterenol (10 nM; β-adrenergic agonist) and/or forskolin (activates adenylyl cyclase to raise intracellular cyclic adenosine monophosphate; cAMP), NPY treatment had no effect on forskolin-induced lipolysis, but increased isoproterenol-induced lipolysis by 30%, suggesting that NPY’s effect occurred upstream of adenylyl cyclase activation [54]. To explain why results differed from previous reports of NPY’s inhibitory effects on lipolysis in cultured adipocytes [14,55,56], it was suggested that NPY’s effect on lipolysis depends on the magnitude of β-adrenergic and lipolytic stimulation by other factors. For example, when concentrations of isoproterenol increased, NPY blunted rather than augmented the stimulation of lipolysis, thus suggesting that perhaps under conditions of strong and weak stimulation of lipolysis, NPY has an inhibitory and stimulatory effect, respectively [54]. Consistent with other studies, the effects of NPY on lipolysis were shown to occur through NPYR1, and it was suggested that differential effects of NPY on lipolysis occurring through the same receptor are due to differences in receptor coupling to different secondary messengers, with inhibitory and stimulatory effects on lipolysis occurring through decreases in cAMP and increases in calcium, respectively [54]. That NPY and NE are co-stored and secreted by postsympathetic nerve terminals in adipose tissue provides an additional layer of complexity to the understanding of how the different systems interact to regulate energy metabolism in adipose tissue [54]. Thus, NPY’s effects on lipolysis can be modulated by nutritional status, adrenergic activity, and changes in receptor activity to achieve tight regulation of energy balance based on energy demand, with differences between visceral and subcutaneous fat.

Thus, NPY’s effects on adipose tissue appear to be related to SNS output and as described above, NPY may influence angiogenesis, adipogenesis, lipolysis, and hypertrophy in WAT. Obesity is characterized by WAT hypercellularity and hypertrophy, particularly in visceral fat, and changes in SNS activity, consistent with enhanced lipid storage and reduced oxidation [57,58]. The decreased SNS outflow observed in some obesity models may stimulate WAT hyperplasia, based on experiments showing that sympathetic nerve denervation induces cellular proliferation in adipose tissue and NE treatment in cell culture reduced preadipocyte proliferation, an effect that was blunted by the β-adrenoceptor antagonist propranolol [59,60]. Although mechanisms of NPY’s role in hyperplasia are not as well studied, it was shown that through NPYR1, NPY stimulated mouse and rat preadipocyte proliferation via activation of the extracellular signal-regulated kinase (ERK) 1/2 signaling pathway [33]. In high-fat diet-fed mice that were exposed to cold stress for 2 weeks, there was an increase in the number of small adipocytes (<10 μM) that were immunoreactive for both NPYR2 and cell proliferation markers, suggesting that NPY plays a role in inducing hyperplasia via NPYR2. Similarly, co-culture of 3 T3-L1 preadipocytes or endothelial cells with sympathetic neuron-derived tumor cells (tyrosine hydroxylase-positive) up-regulated expression of NPYR2 and induced proliferation in both the endothelial cells and preadipocytes, and enhanced differentiation of preadipocytes into adipocytes [30]. Enhanced differentiation was associated with increased lipid accumulation and secretion of leptin and resistin. These effects were blocked by treatment with a NPYR2 receptor antagonist, suggesting that in adipose tissue, SNS-derived NPY modulates proliferation, adipogenesis and angiogenesis via up-regulation of NPYR2 [30].

The SNS innervation to WAT is known to play three major functions including the regulation of lipolysis, cellular proliferation and protein/peptide secretion [47]. Catecholamines (especially NE) are potent lipolytic factors acting through β-adrenergic receptors, which then activate the cAMP – protein kinase A (PKA) signaling cascades. Sympathetic neuron and adipocyte co-culture studies indicated that NPY secreted from sympathetic neurons inhibited β-adrenergic-mediated lipolysis [44], although as discussed above, NPY treatment could elicit different effects on lipolysis depending on the combination of other factors present in the cell culture model [54]. Cross-talk between adipocytes and SNS neurons are thus mediated by multiple signals and NPY may modulate β-adrenoceptor-mediated lipolysis and adipokine secretion. Surgical sympathetic nerve denervation increased the numbers of bromodeoxyuridine-labeled cells that were also immunoreactive for a preadipocyte-specific membrane protein 3 (AD-3), indicating a specific increase in preadipocyte proliferation [61,62]. Decreased sympathetic drive to WAT resulted in WAT expansion that was associated with decreases and increases in β-adrenergic and α_2_-adrenergic receptor numbers, respectively [63].

An in vitro study demonstrated that epinephrine (EPI) enhanced the expression of NPY and its receptors in murine embryonic stem cells (mESCs), and that accelerated differentiation of mESCs into adipocytes was associated with increased expression of preadipocyte factor 1 (PREF-1), fatty acid-binding protein 4 (FABP4) and peroxisome proliferator-activated receptor γ (PPARγ) [64]. These effects were blocked by treatment with NPYR1, 2 and 5 antagonists [64]. The effect of EPI-mediated NPY up-regulation was believed to be associated with greater DNA methylation at the nerve growth factor responsive element and calmodulin-responsive element sites of the NPY gene promoter region [64]. While cell culture-based studies have shown a strong effect of EPI on lipolysis, it has been demonstrated in-vivo that adrenal medullary-derived EPI likely is a minor contributor to whole-body adipose lipolysis, with the majority controlled by SNS-derived NE, as reviewed by [65].

### NPY reduces brown adipose tissue deposition and activation

Brown adipose tissue is almost exclusively under SNS innervation. The release of norepinephrine (NE) from SNS terminals stimulates β_3_-adrenergic receptor-activated BAT thermogenesis [66]. Central administration of NPY in rats inhibited BAT thermogenesis through guanosine diphosphate binding reduction (an indicator of brown fat thermogenic activity) to BAT mitochondria, and stimulated WAT lipid storage by enhancing lipoprotein lipase (LPL) activity, which is a rate-limiting step in catalyzing hydrolysis of plasma lipoproteins into free fatty acids for uptake into peripheral tissues [67]. Despite ample evidence that NPY reduces BAT-associated thermogenesis, it was not until recently that our understanding of the involvement of various CNS-specific nuclei/subnuclei was revealed. Chao et al. demonstrated the role of hypothalamic dorsomedial NPY in adipose tissue function [68]. Knockdown of NPY expression using adeno-associated virus-mediated RNAi in the dorsomedial nucleus (DMN) of rat hypothalamus promoted development of brown adipocytes in inguinal white adipose tissue or transformation from WAT to BAT (also known as brown-in-white, beige or brite cells) characterized by increases in mitochondrial UCP1 and peroxisome proliferator activated receptor-γ coactivator −1 α (PGC1α) expression, when measured at 16 weeks post treatment. This led to increased BAT activity and thereby enhanced energy expenditure and cold-induced thermogenesis [68]. The inducible nature of brown adipocytes in white adipose tissue is intriguing as a possible anti-obesity target and these data show that effects of hypothalamic NPY on brown fat include both inhibition of brown fat thermogenesis and effects on recruitment of brown adipocytes within white adipose depots. These studies are also fascinating because they provide more insight into the physiological function of specific hypothalamic nuclei, such as the DMN.

Other studies using mouse models in which NPY was either overproduced in the ARC of wild type mice or selectively reintroduced into the ARC of otherwise NPY-deficient mice, together with NPY receptor knockout mice, indicated that overexpression of ARC NPY reduced sympathetic outflow via NPYR1 receptor-mediated reduction in tyrosine hydroxylase (TH; an indicator of SNS outflow) expression in the PVN and various regions in the brainstem. Reduced SNS innervation was associated with the down-regulation of UCP1 expression in BAT, which could be reversed after surgical sympathetic denervation to BAT [69]. The ICV injection of NPY suppressed SNS activity in a dose-dependent manner, which was followed by a gradual recovery. Unilaterally microinjecting NPY into the paraventricular nucleus (PVN) suppressed the SNS, and the opposite was observed after medial preoptic area microinjection. No effect was observed with injection into the anterior hypothalamic area, ventromedial nucleus (VMN), or lateral hypothalamus (LH) [70]. Reduced SNS outflow decreases release of NE from sympathetic nerve endings and inhibits the thermogenic function of brown adipose tissue (BAT) by deactivating the cAMP-dependent PKA pathway, which further down-regulates UCP1-associated thermogenesis.Taken together, these data indicate that NPY promotes positive energy balance by stimulating adipogenesis and inhibiting lipolysis in WAT. Increased thermogenesis in brown fat and recruitment of brown adipocytes in white adipose tissue after NPY suppression suggests that the NPY system also has an inhibitory effect on BAT activity. These effects appear to be mediated through the regulation of the hypothalamus-SNS-adipose tissue axis. The possible mechanisms described above are summarized in Figures 1 and 2.

**Figure 1:** **Antilipolytic and adipogenic effects of NPY on white adipose tissue.** In the peripheral system, NPY binds to receptors 1, 2 and 5 and affects β-adrenergic receptor (β_1_-AR, β_2_-AR and β_3_-AR; mainly through β_2_-AR) configuration, the modification thereby leading to improved affinity for Gαi proteins. Subsequently, this activation of inhibitory GTP-binding protein alpha subunit (Gαi) inhibits adenylyl cyclase (AC) and cyclic AMP (cAMP) production. Decreased cellular cAMP levels inhibit protein kinase A (PKA), which phosphorylates and activates hormone-sensitive lipase (HSL). Decreased PKA activity also inhibits phosphorylation of lipid droplet-associated protein perilipin (peri) into PeriA, which controls the magnitude of lipolysis. Lipolysis is catalyzed by 3 lipases. Triacylglycerol is firstly hydrolyzed by adipocyte triglyceride lipase (ATGL) resulting in the formation of diacylglycerol (DAG) and release of a fatty acid (FA). Monoacylglycerol lipase (MGL) catalyzes hydrolysis of MAG, yielding glycerol and a FA. Increased hypothalamic (abbreviated as hypo in the figure) NPY inhibits sympathetic nerve system (SNS) outflow and suppresses catecholamine release, mainly norepinephrine (NE), and thereby their binding to β-adrenergic receptors, which in turn reduces the cAMP-PKA pathway-associated lipolysis. On the other hand, NPY itself in the peripheral system can stimulate ERK-mediated adipogenesis. Through the hypothalamus-SNS-adipose tissue axis, reduced NE enhances adipogenesis via undefined mechanisms. Reduced SNS outflow is compensated for by adrenal medullary catecholamines, primarily epinephrine (EPI), which was also known to stimulate adipogenesis, possibly through NPY regulation. Parts of the figure are adapted from references [71,72]. “**→**”: stimulatory effect; “**⊣**”: inhibitory effect ;“**······›**”mechanisms unknown; “**─··─·›**” compensatory effect of EPI secretion.

**Figure 2:** **NPY inhibits BAT thermogenesis via reduced SNS outflow.** Increased release of NPY in the hypothalamus inhibits sympathetic nerve system (SNS) outflow, particularly norepinephrine (NE) release. Consequently, it inhibits the cAMP-PKA signaling pathway via β-adrenergic receptors. Reduced lipolysis decreases the level of fatty acid storage in the brown adipose tissue, together with reduced uncoupling protin 1 (UCP1) expression and secretion, resulting in reduced thermogenic potential. Consequently, with less fatty acids being transported into the mitochondria by the carnitine palmitoyl transferase (carnitine shuttle) and also reduced UCP1 functioning to dissipate the proton-motive force across the mitochondrial membrane, there is less heat production. Part of the picture is summarized from [73].

### Hypothalamus-adipose tissue crosstalk

The NPY system represents a form of communication between the hypothalamus and adipose tissue, and is linked to positive energy balance through increases in energy intake and storage and reduced energy expenditure. This is achieved indirectly through bidirectional neuronal and hormonal communication, and possibly via direct circulation through the blood brain barrier. The hypothalamus is the energy sensory center for signals produced by peripheral tissues such as the gastrointestinal tract and adipose tissue. Hypothalamus-mediated white and brown adipose tissue turnover is mainly regulated through SNS outflow, as summarized above. The study of the role of specific hypothalamic nuclei in the regulation of peripheral adiposity did not receive much attention until recently, partly due to advents in molecular technology as well as a better understanding of brain neural circuits. A body of evidence has shown that NPY in the ARC, PVN, and DMN neurons is involved in adiposity and BAT thermogenesis through regulation of the SNS outflow [68,69]. Whether other hypothalamic nuclei play the same role remains elusive.

While early studies revealed that adipose tissue was innervated by the sympathetic nervous system, they did not reveal the specific brain nuclei from which the SNS outflow to WAT originated. A transneuronal tract tracer, a pseudorabies virus (PRV), was used for this purpose, because it is a neurotropic virus that binds to the presynaptic neural membrane, fuses with the axon membrane, and then delivers uncoated capsids in the axon (described in an excellent review by [47]). The capsids are then transported to the cell body where they replicate and can exit the infected cell via the dendrites, thereby only infecting neurons that are synaptically connected to those PRV-containing cells [47]. Immunostaining after PRV injection into fat revealed that in hamsters, regions of the hypothalamus including the ARC, dorsal, lateral, suprachiasmatic, PVN, and nuclei and medial preoptic area, were identified as sites that modulated SNS outflow to the WAT [47]. Hypothalamus-SNS-BAT circuitries were demonstrated to be hyperactive in the PVN, DMN, LH, anterior hypothalamic nucleus, and posterior hypothalamic nucleus [74]. Whether adipose tissue is also under the control of the parasympathetic nervous system is still controversial [75,76]. Identification of hypothalamic nuclei associated with adiposity and brown fat thermogenesis may provide better targets toward the control of overweight and obesity through the manipulation of the hypothalamus-adipose tissue axis, and allow for development of more pathway-specific therapeutic strategies.

Adipose tissue not only dynamically accumulates and releases lipids, but also serves as an endocrine organ that produces adipokines, hormones, and appetite-regulating factors as the sensory input reflecting the amount of lipid and adipocyte turnover. Sensory information is transported via dorsal root ganglion to the spinal cord and then on to the brain to interact with the SNS outflow to the adipose tissue [47,74,77]. The sensory innervation of adipose tissue may serve as a feedback loop to regulate the level of its sympathetic drive and also regulate adipocyte turnover [78]. Sensory information includes adipokines such as adiponectin, apelin, resistin and leptin, that all target various regions in the hypothalamus and regulate body energy homeostasis [79]. Leptin is one of the best studied adipokines that informs the brain of body fat levels. Treatment of human abdominal subcutaneous adipocytes with recombinant human NPY reduced leptin secretion but did not affect release of adiponectin and tumor necrosis factor α [31]. Interestingly, high fat diet-induced diabetic mice subjected to intra-abdominal UCP1 overexpression using an adenoviral vector had significantly reduced food intake characterized by reduced NPY mRNA in the hypothalamus, and improved insulin and leptin sensitivity. Local nerve dissection showed that these actions were achieved by afferent-nerve signals from intra-abdominal fat tissue to the hypothalamus that modulated hypothalamic leptin sensitivity, illustrating the importance of the hypothalamus-adipose tissue feedback loop [80]. This may suggest that brown adipocytes in WAT play an important role in whole-body energy metabolism and ectopic UCP1 expression could be a promising future research direction. In summary, an adiposity negative-feedback model indicates that adiposity signals can inform the brain of changes in body fat mass so that the brain can mount adaptive adjustments in energy intake to stabilize fat stores in the long term. Understanding the neural signaling pathways and endocrine regulation associated with the adiposity negative feedback may provide a new avenue for treatment of obesity and associated diseases.

### Central vs. peripheral circulating NPY

NPY is expressed in both the hypothalamus and periphery and is detected in the circulation. Understanding the cellular sources, routes of delivery to various tissues and the rate of decay are critical for understanding the physiological roles of NPY. The majority of NPY is secreted by the neurons in the CNS with lower concentrations in the peripheral system. In the SVF fraction of adipose tissue from mice, secreted NPY was reported to be in the picomolar range, consistent with physiological concentrations in humans [29]. Recent studies showed that the concentration of cerebrospinal fluid (CSF) NPY (cNPY; 792.1 pg/mL) was 3 fold greater than plasma NPY (pNPY; 220.0 pg/mL) in humans [81]. Therefore, whether hypothalamus-derived NPY can enter the blood stream is critical in understanding the regulation of food intake and fat deposition. A clinical study demonstrated that circulating NPY in obese women was elevated as compared to women from the control group [82]. However, no statistically significant cross-correlations have been identified between CSF and plasma NPY in healthy males. Circulating NPY was also elevated in genetically obese mice [30]. The cNPY/pNPY ratio depends on the rates of NPY production, degradation, reabsorbtion in both compartments and potential transport across the blood brain barrier. Although NPY was shown to cross the blood–brain barrier intact via a non-saturatable transporter in rats, which is still unidentified in humans [83], the absence of cross-correlation between CSF and plasma may be due to local protease degradation as indicated by Baker et al. [52]. As a peptide, the active window of time for NPY is short as compared to a steroid neurotransmitter. Ahlborg et al. showed that in adult men the half-life for NPY is up to 39 min [84]. The concentration of NPY in both central and peripheral compartments has a higher heritability than other neuropeptides [85,86], which makes it an attractive candidate for research on genetic aspects of metabolic diseases. Thus, a further understanding of factors governing NPY concentrations and transport in the circulation and between central and peripheral systems, especially in humans, will rely on more research together with advanced techniques that are sensitive to lower concentrations of NPY.

## Conclusions and implications

Neuropeptide Y stimulates food intake and white fat deposition and at the same time reduces brown fat activation and consequently thermogenesis, yielding a net accumulation of energy via enhanced energy intake and storage (Figure 3). The function of NPY is determined by site-specific NPY and NPY receptor-subtype expression, NPY release, degradation, and concentrations in the circulation, all of which are regulated by numerous energy balance strategies. This provides tight regulation of an essential system to ensure that the NPY signals can respond rapidly and for prolonged durations during short and long-term control of energy homeostasis in various food-accessible conditions. Understanding the role of NPY in energy homeostasis has critical implications for biomedical applications, the most common pharmacological therapies nowadays for obesity involving gastrointestinal surgery and pharmacological interventions. Drugs that are intended for weight loss affect either metabolism by reducing absorption of nutrients from food or through the CNS by decreasing appetite and increasing energy expenditure. In light of the purported systemic role of NPY, it becomes a promising candidate for controlling the development and treatment of obesity. Whether NPY can be used as a biomarker for obesity awaits further determination. A body of studies aimed to manipulate NPY and NPY receptor-subtype function highlight the feasibility of targeting the NPY system for therapeutic strategies. However, the mechanisms underlying the effects of NPY are complicated, especially in view of brain-adipose cross talk.

**Figure 3:** **Role of NPY in energy intake and expenditure.** cNPY: NPY in the central nervous system; pNPY: Peripheral NPY; BBB: Blood brain barrier; Hypo: hypothalamus. The cNPY stimulates food intake mainly via NPYR1 and NPYR5 to increase energy intake. Additionally, through the hypothalamus-SNS-adipose axis, NPY reduces sympathetic nervous system (SNS) outflow, which promotes white adipose tissue (WAT) deposition by enhancing adipogenesis and inhibiting lipolysis, as well as inhibiting brown adipose tissue (BAT) deposition and associated nonshivering thermogenesis. The same effects in WAT were achieved by peripheral NPY via different signaling pathways. This collectively leads to energy storage in adipose tissue. Adipose-hypothalamus crosstalk serves as a feedback loop via sensory inflow that informs the brain of the long-term peripheral energy status so that the brain can make the necessary adjustment. Numerous adipokines, hormones, and appetite regulating factors have been identified that play an important role in adjusting energy balance through the hypothalamus either by directly affecting food intake or regulating adiposity through SNS outflow, such as leptin, NPY, and UCP1. NPY is more abundant in the central nervous system as compared to the peripheral system. Whether and how it crosses the blood brain barrier is critical for understanding its role in energy regulation.

## Abbreviations

AD-3: Pre-adipocyte membrane protein 3; AgRP: Agouti-related peptide; ARC: Arcuate nucleus of the hypothalamus; BAT: Brown adipose tissue; cAMP: Cyclic adenosine monophosphate; CNS: Central nervous system; DMN: Dorsomedial nucleus; EPI: Epinephrine; ERK: Extracellular signal-regulated kinase; FABP4: Fatty acid-binding protein 4; ICV: Intracerebroventricular; LH: Lateral hypothalamus; LPL: Lipoprotein lipase; MC3R: Melanocortin receptor 3; MC4R: Melanocortin receptor 4; NPYR: Neuropeptide Y receptor; NPY: Neuropeptide Y; NPYR1: Neuropeptide Y receptor sub-type 1; NPYR2: Neuropeptide Y receptor sub-type 2; NPYR5: Neuropeptide Y receptor sub-type 5; NE: Norepinephrine; OHDA: 6-hydroxydopamine; PGC1α: Peroxisome proliferator activated receptor-γ coactivator −1 α; PKA: Protein kinase A; PPARγ: Peroxisome proliferator-activated receptor γ; PREF-1: Preadipocyte factor 1; PRV: Pseudorabies virus; PVN: Paraventricular nucleus; SVF: Stromal-vascular fraction; SNS: Sympathetic nervous system; TAG: Triacylglycerol; TH: Tyrosine hydroxylase; UCP1: Uncoupling protein 1; VMN: Ventromedial nucleus; WAT: White adipose tissue.

## Competing interests

There are no competing interests to disclose for any of the authors.

## Authors’ contributions

WZ contributed to the literature search, synthesis of information and preparation of the manuscript. MAC and ERG reviewed, edited and revised the final version. All authors had final approval of the submitted version.

## References

[B1] MortonGJCummingsDEBaskinDGBarshGSSchwartzMWCentral nervous system control of food intake and body weightNature20064432892951698870310.1038/nature05026

[B2] RosenEDSpiegelmanBMAdipocytes as regulators of energy balance and glucose homeostasisNature20064448478531716747210.1038/nature05483PMC3212857

[B3] MercerRECheeMJColmersWFThe role of NPY in hypothalamic mediated food intakeFront Neuroendocrinol2011323984152172657310.1016/j.yfrne.2011.06.001

[B4] CarlquistMJornvallHTatemotoKMuttVA porcine brain polypeptide is identical to the vasoactive intestinal polypeptideGastroenterology1982832452497084607

[B5] GeorgeMRajaramMShanmugamENew and emerging drug molecules against obesityJ Cardiovasc Pharmacol Ther20141965762406400910.1177/1074248413501017

[B6] BrobergerCJohansenJJohanssonCSchallingMHokfeltTThe neuropeptide Y/agouti gene-related protein (AGRP) brain circuitry in normal, anorectic, and monosodium glutamate-treated miceProc Natl Acad Sci U S A1998951504315048984401210.1073/pnas.95.25.15043PMC24572

[B7] KohnoDYadaTArcuate NPY neurons sense and integrate peripheral metabolic signals to control feedingNeuropeptides2012463153192310736510.1016/j.npep.2012.09.004

[B8] LeibowitzSFWortleyKEHypothalamic control of energy balance: different peptides, different functionsPeptides2004254735041513486810.1016/j.peptides.2004.02.006

[B9] LarhammarDBlomqvistAGSoderbergCEvolution of neuropeptide Y and its related peptidesComp Biochem Physiol C1993106743752790581010.1016/0742-8413(93)90236-e

[B10] NaveilhanPNeveuIArenasEErnforsPComplementary and overlapping expression of Y1, Y2 and Y5 receptors in the developing and adult mouse nervous systemNeuroscience199887289302972215810.1016/s0306-4522(98)00141-9

[B11] GehlertDRRole of hypothalamic neuropeptide Y in feeding and obesityNeuropeptides1999333293381065751010.1054/npep.1999.0057

[B12] BatterhamRLCowleyMASmallCJHerzogHCohenMADakinCLWrenAMBrynesAELowMJGhateiMAConeRDBloomSRGut hormone PYY(3–36) physiologically inhibits food intakeNature20024186506541216786410.1038/nature00887

[B13] KamijiMMInuiANeuropeptide y receptor selective ligands in the treatment of obesityEndocr Rev2007286646841778542710.1210/er.2007-0003

[B14] LabelleMBoulangerYFournierASt PierreSSavardRTissue-specific regulation of fat cell lipolysis by NPY in 6-OHDA-treated ratsPeptides199718801808928592810.1016/s0196-9781(97)00028-4

[B15] IshiharaATanakaTKanataniAFukamiTIharaMFukurodaTA potent neuropeptide Y antagonist, 1229U91, suppressed spontaneous food intake in Zucker fatty ratsAm J Physiol1998274R1500R1504961242010.1152/ajpregu.1998.274.5.R1500

[B16] KanataniAIshiharaAAsahiSTanakaTOzakiSIharaMPotent neuropeptide Y Y1 receptor antagonist, 1229U91: blockade of neuropeptide Y-induced and physiological food intakeEndocrinology199613731773182875473610.1210/endo.137.8.8754736

[B17] MullinsDKirbyDHwaJGuzziMRivierJParkerEIdentification of potent and selective neuropeptide Y Y(1) receptor agonists with orexigenic activity in vivoMol Pharmacol20016053454011502885

[B18] BurcelinRBrunnerHSeydouxJThorensaBPedrazziniTIncreased insulin concentrations and glucose storage in neuropeptide Y Y1 receptor-deficient micePeptides2001224214271128709710.1016/s0196-9781(01)00357-6

[B19] KushiASasaiHKoizumiHTakedaNYokoyamaMNakamuraMObesity and mild hyperinsulinemia found in neuropeptide Y-Y1 receptor-deficient miceProc Natl Acad Sci U S A1998951565915664986102610.1073/pnas.95.26.15659PMC28100

[B20] BalasubramaniamAJoshiRSuCFriendLAJamesJHNeuropeptide Y (NPY) Y2 receptor-selective agonist inhibits food intake and promotes fat metabolism in mice: combined anorectic effects of Y2 and Y4 receptor-selective agonistsPeptides2007282352401720434910.1016/j.peptides.2006.08.041

[B21] SainsburyASchwarzerCCouzensMFetissovSFurtingerSJenkinsACoxHMSperkGHokfeltTHerzogHImportant role of hypothalamic Y2 receptors in body weight regulation revealed in conditional knockout miceProc Natl Acad Sci U S A200299893889431207256210.1073/pnas.132043299PMC124402

[B22] SainsburyASchwarzerCCouzensMJenkinsAOakesSROrmandyCJHerzogHY4 receptor knockout rescues fertility in ob/ob miceGenes Dev200216107710881200079110.1101/gad.979102PMC186243

[B23] SchaffhauserAOStricker-KrongradABrunnerLCuminFGeraldCWhitebreadSCriscioneLHofbauerKGInhibition of food intake by neuropeptide Y Y5 receptor antisense oligodeoxynucleotidesDiabetes19974617921798935602810.2337/diab.46.11.1792

[B24] Tang-ChristensenMKristensenPStidsenCEBrandCLLarsenPJCentral administration of Y5 receptor antisense decreases spontaneous food intake and attenuates feeding in response to exogenous neuropeptide YJ Endocrinol1998159307312979537210.1677/joe.0.1590307

[B25] MarshDJHollopeterGKaferKEPalmiterRDRole of the Y5 neuropeptide Y receptor in feeding and obesityNat Med19984718721962398310.1038/nm0698-718

[B26] HirschDZukowskaZNPY and stress 30 years later: the peripheral viewCell Mol Neurobiol2012326456592227117710.1007/s10571-011-9793-zPMC3492947

[B27] LarsenPJKristensenPCentral Y4 receptor distribution. Radioactive ribonucleotide probe in situ hybridization with in vitro receptor autoradiographyMethods Mol Biol20001531851981095799310.1385/1-59259-042-X:185

[B28] LinSShiYCYulyaningsihEAljanovaAZhangLMaciaLNguyenADLinEJDuringMJHerzogHSainsburyACritical role of arcuate Y4 receptors and the melanocortin system in pancreatic polypeptide-induced reduction in food intake in micePLoS One20094e84882004112910.1371/journal.pone.0008488PMC2796177

[B29] SingerKMorrisDLOatmenKEWangTDelPropostoJMergianTChoKWLumengCNNeuropeptide Y is produced by adipose tissue macrophages and regulates obesity-induced inflammationPLoS One20138e579292347212010.1371/journal.pone.0057929PMC3589443

[B30] KuoLEKitlinskaJBTilanJULiLBakerSBJohnsonMDLeeEWBurnettMSFrickeSTKvetnanskyRHerzogHZukowskaZNeuropeptide Y acts directly in the periphery on fat tissue and mediates stress-induced obesity and metabolic syndromeNat Med2007138038111760349210.1038/nm1611

[B31] KosKHarteALJamesSSneadDRO'HareJPMcTernanPGKumarSSecretion of neuropeptide Y in human adipose tissue and its role in maintenance of adipose tissue massAm J Physiol Endocrinol Metab2007293E1335E13401778550110.1152/ajpendo.00333.2007

[B32] SitticharoonCChatreeSChurintaraphanMExpressions of neuropeptide Y and Y1 receptor in subcutaneous and visceral fat tissues in normal weight and obese humans and their correlations with clinical parameters and peripheral metabolic factorsRegul Pept201318565722383811210.1016/j.regpep.2013.06.015

[B33] YangKGuanHAranyEHillDJCaoXNeuropeptide Y is produced in visceral adipose tissue and promotes proliferation of adipocyte precursor cells via the Y1 receptorFASEB J200822245224641832340510.1096/fj.07-100735

[B34] ZhangWSumnersLHSiegelPBClineMAGilbertERQuantity of glucose transporter and appetite-associated factor mRNA in various tissues after insulin injection in chickens selected for low or high body weightPhysiol Genomics201345108410942404627910.1152/physiolgenomics.00102.2013

[B35] GongHXGuoXRFeiLGuoMLiuQQChenRHLipolysis and apoptosis of adipocytes induced by neuropeptide Y-Y5 receptor antisense oligodeoxynucleotides in obese ratsActa Pharmacol Sin20032456957512791184

[B36] Rosmaninho-SalgadoJCortezVEstradaMSantanaMMGoncalvesAMarquesAPCavadasCIntracellular mechanisms coupled to NPY Y2 and Y5 receptor activation and lipid accumulation in murine adipocytesNeuropeptides2012463593662298115910.1016/j.npep.2012.08.006

[B37] GerickeMTKosackaJKochDNowickiMSchroderTRickenAMNieberKSpanel-BorowskiKReceptors for NPY and PACAP differ in expression and activity during adipogenesis in the murine 3T3-L1 fibroblast cell lineBr J Pharmacol20091576206321942240010.1111/j.1476-5381.2009.00164.xPMC2707974

[B38] SethiJKVidal-PuigAJThematic review series: adipocyte biology. Adipose tissue function and plasticity orchestrate nutritional adaptationJ Lipid Res200748125312621737488010.1194/jlr.R700005-JLR200PMC4303760

[B39] KopeckyJClarkeGEnerbackSSpiegelmanBKozakLPExpression of the mitochondrial uncoupling protein gene from the aP2 gene promoter prevents genetic obesityJ Clin Invest19959629142923867566310.1172/JCI118363PMC186003

[B40] LowellBBS-SusulicVHamannALawittsJAHimms-HagenJBoyerBBKozakLPFlierJSDevelopment of obesity in transgenic mice after genetic ablation of brown adipose tissueNature1993366740742826479510.1038/366740a0

[B41] NedergaardJBengtssonTCannonBUnexpected evidence for active brown adipose tissue in adult humansAm J Physiol Endocrinol Metab2007293E444E4521747305510.1152/ajpendo.00691.2006

[B42] CypessAMLehmanSWilliamsGTalIRodmanDGoldfineABKuoFCPalmerELTsengYHDoriaAKolodnyGMKahnCRIdentification and importance of brown adipose tissue in adult humansN Engl J Med2009360150915171935740610.1056/NEJMoa0810780PMC2859951

[B43] KirklandJLDobsonDEPreadipocyte function and aging: links between age-related changes in cell dynamics and altered fat tissue functionJ Am Geriatr Soc199745959967925684910.1111/j.1532-5415.1997.tb02967.x

[B44] TurtzoLCMarxRLaneMDCross-talk between sympathetic neurons and adipocytes in cocultureProc Natl Acad Sci U S A20019812385123901160678210.1073/pnas.231478898PMC60063

[B45] MorrisJLCotransmission from sympathetic vasoconstrictor neurons to small cutaneous arteries in vivoAm J Physiol1999277H58H641040918210.1152/ajpheart.1999.277.1.H58

[B46] LundbergJMFranco-CerecedaAHemsenALacroixJSPernowJPharmacology of noradrenaline and neuropeptide tyrosine (NPY)-mediated sympathetic cotransmissionFundam Clin Pharmacol19904373391217025310.1111/j.1472-8206.1990.tb00692.x

[B47] BartnessTJKay SongCShiHBowersRRFosterMTBrain-adipose tissue cross talkProc Nutr Soc20056453641587792310.1079/pns2004409

[B48] Rosmaninho-SalgadoJMarquesAPEstradaMSantanaMCortezVGrouzmannECavadasCDipeptidyl-peptidase-IV by cleaving neuropeptide Y induces lipid accumulation and PPAR-gamma expressionPeptides20123749542281977310.1016/j.peptides.2012.06.014

[B49] BradleyRLMansfieldJPMaratos-FlierENeuropeptides, including neuropeptide Y and melanocortins, mediate lipolysis in murine adipocytesObes Res2005136536611589747310.1038/oby.2005.73

[B50] KuoLECzarneckaMKitlinskaJBTilanJUKvetnanskyRZukowskaZChronic stress, combined with a high-fat/high-sugar diet, shifts sympathetic signaling toward neuropeptide Y and leads to obesity and the metabolic syndromeAnn N Y Acad Sci200811482322371912011510.1196/annals.1410.035PMC2914537

[B51] ShiYCLinSCastilloLAljanovaAEnriquezRFNguyenADBaldockPAZhangLBijkerMSMaciaLYulyaningsihEZhangHLauJSainsburyAHerzogHPeripheral-specific y2 receptor knockdown protects mice from high-fat diet-induced obesityObesity (Silver Spring)201119213721482154693010.1038/oby.2011.99

[B52] BakerSBCohenMKuoLJohnsonMAl-AttarAZukowskaZThe role of the neuropeptide Y2 receptor in liporemodeling: neuropeptide Y-mediated adipogenesis and adipose graft maintenancePlast Reconstr Surg20091234864921918260510.1097/PRS.0b013e3181954c80PMC2659679

[B53] NguyenNLRandallJBanfieldBWBartnessTJCentral Sympathetic Innervations to Visceral and Subcutaneous White Adipose TissueAm J Physiol Regul Integr Comp Physiol201430637538610.1152/ajpregu.00552.2013PMC394910724452544

[B54] LiRGuanHYangKNeuropeptide Y potentiates beta-adrenergic stimulation of lipolysis in 3 T3-L1 adipocytesRegul Pept201217816202275027710.1016/j.regpep.2012.06.002

[B55] ValetPBerlanMBeauvilleMCrampesFMontastrucJLLafontanMNeuropeptide Y and peptide YY inhibit lipolysis in human and dog fat cells through a pertussis toxin-sensitive G proteinJ Clin Invest199085291295210488010.1172/JCI114425PMC296417

[B56] CastanIValetPQuideauNVoisinTAmbidLLaburtheMLafontanMCarpeneCAntilipolytic effects of alpha 2-adrenergic agonists, neuropeptide Y, adenosine, and PGE1 in mammal adipocytesAm J Physiol1994266R1141R1147791043410.1152/ajpregu.1994.266.4.R1141

[B57] HausmanDBDiGirolamoMBartnessTJHausmanGJMartinRJThe biology of white adipocyte proliferationObes Rev200122392541211999510.1046/j.1467-789x.2001.00042.x

[B58] BrayGAObesity–a state of reduced sympathetic activity and normal or high adrenal activity (the autonomic and adrenal hypothesis revisited)Int J Obes199014Suppl 37791discussion 91–722086518

[B59] FosterMTBartnessTJSympathetic but not sensory denervation stimulates white adipocyte proliferationAm J Physiol Regul Integr Comp Physiol2006291R1630R16371688792110.1152/ajpregu.00197.2006

[B60] GeloenAColletAJBukowieckiLJRole of sympathetic innervation in brown adipocyte proliferationAm J Physiol1992263R1176R1181148192410.1152/ajpregu.1992.263.6.R1176

[B61] WrightJTHausmanGJMonoclonal antibodies against cell surface antigens expressed during porcine adipocyte differentiationInt J Obes1990143954092384293

[B62] KrasKMHausmanDBHausmanGJMartinRJAdipocyte development is dependent upon stem cell recruitment and proliferation of preadipocytesObes Res199974914971050960710.1002/j.1550-8528.1999.tb00438.x

[B63] CarpeneCRebourcetMCGuichardCLafontanMLavauMIncreased alpha 2-adrenergic binding sites and antilipolytic effect in adipocytes from genetically obese ratsJ Lipid Res1990318118192166122

[B64] HanRKitlinskaJBMundayWRGallicanoGIZukowskaZStress hormone epinephrine enhances adipogenesis in murine embryonic stem cells by up-regulating the neuropeptide Y systemPLoS One20127e366092257073110.1371/journal.pone.0036609PMC3343033

[B65] BartnessTJSongCKThematic review series: adipocyte biology. Sympathetic and sensory innervation of white adipose tissueJ Lipid Res200748165516721746032710.1194/jlr.R700006-JLR200

[B66] BartnessTJSongCKInnervation of brown adipose tissue and its role in thermogenesisCanadian Journal of Diabetes2005299

[B67] BillingtonCJBriggsJEGraceMLevineASEffects of intracerebroventricular injection of neuropeptide Y on energy metabolismAm J Physiol1991260R321R327199671910.1152/ajpregu.1991.260.2.R321

[B68] ChaoPTYangLAjaSMoranTHBiSKnockdown of NPY expression in the dorsomedial hypothalamus promotes development of brown adipocytes and prevents diet-induced obesityCell Metab2011135735832153133910.1016/j.cmet.2011.02.019PMC3093161

[B69] ShiYCLauJLinZZhangHZhaiLSperkGHeilbronnRMietzschMWegerSHuangXFEnriquezRFBaldockPAZhangLSainsburyAHerzogHLinSArcuate NPY controls sympathetic output and BAT function via a relay of tyrosine hydroxylase neurons in the PVNCell Metab2013172362482339517010.1016/j.cmet.2013.01.006

[B70] EgawaMYoshimatsuHBrayGANeuropeptide Y suppresses sympathetic activity to interscapular brown adipose tissue in ratsAm J Physiol1991260R328R334199672010.1152/ajpregu.1991.260.2.R328

[B71] AltarejosJYMontminyMCREB and the CRTC co-activators: sensors for hormonal and metabolic signalsNat Rev Mol Cell Biol2011121411512134673010.1038/nrm3072PMC4324555

[B72] JaworskiKSarkadi-NagyEDuncanREAhmadianMSulHSRegulation of triglyceride metabolism. IV. Hormonal regulation of lipolysis in adipose tissueAm J Physiol Gastrointest Liver Physiol2007293G1G41721847110.1152/ajpgi.00554.2006PMC2887286

[B73] TownsendKTsengYHBrown adipose tissue: recent insights into development, metabolic function and therapeutic potentialAdipocyte2012113242370050710.4161/adip.18951PMC3661118

[B74] LiuYNeural Crosstalk between Sympathetic Nervous System and Sensory Circuits to Brown Adipose Tissue, Thesis2013Department of Biology: Georgia State University135

[B75] BartnessTJSongCKBrain-adipose tissue neural crosstalkPhysiol Behav2007913433511752168410.1016/j.physbeh.2007.04.002PMC1986714

[B76] BartnessTJDual innervation of white adipose tissue: some evidence for parasympathetic nervous system involvementJ Clin Invest2002110123512371241756010.1172/JCI17047PMC151621

[B77] SongCKSchwartzGJBartnessTJAnterograde transneuronal viral tract tracing reveals central sensory circuits from white adipose tissueAm J Physiol Regul Integr Comp Physiol2009296R501R5111910936710.1152/ajpregu.90786.2008PMC2665851

[B78] RalevicVKaroonPBurnstockGLong-term sensory denervation by neonatal capsaicin treatment augments sympathetic neurotransmission in rat mesenteric arteries by increasing levels of norepinephrine and selectively enhancing postjunctional actionsJ Pharmacol Exp Ther199527464717616449

[B79] YiCXTschopMHBrain-gut-adipose-tissue communication pathways at a glanceDis Model Mech201255835872291501910.1242/dmm.009902PMC3424454

[B80] YamadaTKatagiriHIshigakiYOgiharaTImaiJUnoKHasegawaYGaoJIshiharaHNiijimaAManoHAburataniHAsanoTOkaYSignals from intra-abdominal fat modulate insulin and leptin sensitivity through different mechanisms: neuronal involvement in food-intake regulationCell Metab200632232291651740910.1016/j.cmet.2006.02.001

[B81] BakerDGBertramTMPatelPMBarkauskasDACloptonPPatelSGeraciotiTDJrHajiUO'ConnorDTNievergeltCMHaugerRLCharacterization of cerebrospinal fluid (CSF) and plasma NPY levels in normal volunteers over a 24-h timeframePsychoneuroendocrinology201338237823822375933410.1016/j.psyneuen.2013.04.020

[B82] BaranowskaBWolinska-WitortEMartynskaLChmielowskaMMazurczak-PlutaTBoguradzkaABaranowska-BikASibutramine therapy in obese women–effects on plasma neuropeptide Y (NPY), insulin, leptin and beta-endorphin concentrationsNeuro Endocrinol Lett20052667567916380708

[B83] KastinAJAkerstromVNonsaturable entry of neuropeptide Y into brainAm J Physiol1999276E479E4821007001310.1152/ajpendo.1999.276.3.E479

[B84] AhlborgGWeitzbergESolleviALundbergJMSplanchnic and renal vasoconstrictor and metabolic responses to neuropeptide Y in resting and exercising manActa Physiol Scand1992145139149163644310.1111/j.1748-1716.1992.tb09349.x

[B85] ZhangKRaoFMiramontes-GonzalezJPHightowerCMVaughtBChenYGreenwoodTASchorkAJWangLMahataMStridsbergMKhandrikaSBiswasNFungMMWaalenJMiddelbergRPHeathACMontgomeryGWMartinNGWhitfieldJBBakerDGSchorkNJNievergeltCMO'ConnorDTNeuropeptide Y (NPY): genetic variation in the human promoter alters glucocorticoid signaling, yielding increased NPY secretion and stress responsesJ Am Coll Cardiol201260167816892302133310.1016/j.jacc.2012.06.042PMC3687554

[B86] BerrettiniWHOxenstiernaGSedvallGNurnbergerJIJrGoldPWRubinowDRGoldinLRCharacteristics of cerebrospinal fluid neuropeptides relevant to clinical researchPsychiatry Res198825349359318686310.1016/0165-1781(88)90104-7

